# miR-335 Targets LRRK2 and Mitigates Inflammation in Parkinson’s Disease

This article has been retracted.

**DOI:** 10.3389/fcell.2021.661461

**Published:** 2021-06-15

**Authors:** Sara R. Oliveira, Pedro A. Dionísio, Maria M. Gaspar, Leonor Correia Guedes, Miguel Coelho, Mário M. Rosa, Joaquim J. Ferreira, Joana D. Amaral, Cecília M. P. Rodrigues

**Affiliations:** ^1^Research Institute for Medicines (iMed.ULisboa), Faculty of Pharmacy, Universidade de Lisboa, Lisbon, Portugal; ^2^Instituto de Medicina Molecular João Lobo Antunes, Faculdade de Medicina, Universidade de Lisboa, Lisbon, Portugal; ^3^Department of Neuroscience and Mental Health, Neurology, Hospital de Santa Maria, Centro Hospitalar Universitário Lisboa Norte, Lisbon, Portugal; ^4^Laboratory of Clinical Pharmacology and Therapeutics, Faculdade de Medicina, Universidade de Lisboa, Lisbon, Portugal

**Keywords:** inflammation, LRRK2, miR-335, necroptosis, Parkinson’s disease

## Abstract

Parkinson’s disease (PD) is mainly driven by dopaminergic neuronal degeneration in the *substantia nigra pars compacta* accompanied by chronic neuroinflammation. Despite being mainly sporadic, approximately 10% of all cases are defined as heritable forms of PD, with mutations in the leucine-rich repeat kinase (*LRRK2*) gene being the most frequent known cause of familial PD. MicroRNAs (miRNAs or miRs), including miR-335, are frequently deregulated in neurodegenerative diseases, such as PD. Here, we aimed to dissect the protective role of miR-335 during inflammation and/or neurodegenerative events in experimental models of PD. Our results showed that miR-335 is significantly downregulated in different PD-mimicking conditions, including BV2 microglia cells stimulated with lipopolysaccharide (LPS) and/or overexpressing wild-type LRRK2. Importantly, these results were confirmed in serum of mice injected with 1-methyl-1-4-phenyl-1,2,3,6-tetrahydripyridine hydrochloride (MPTP), and further validated in patients with idiopathic PD (iPD) and those harboring mutations in *LRRK2* (LRRK2-PD), thus corroborating potential clinical relevance. Mechanistically, miR-335 directly targeted LRRK2 mRNA. In the BV2 and N9 microglia cell lines, miR-335 strongly counteracted LPS-induced proinflammatory gene expression, and downregulated receptor interacting protein 1 (RIP1) and RIP3, two important players of necroptotic and inflammatory signaling pathways. Further, miR-335 inhibited LPS-mediated ERK1/2 activation. LRRK2-Wt-induced proinflammatory gene expression was also significantly reduced by miR-335 overexpression. Finally, in SH-SY5Y neuroblastoma cells, miR-335 decreased the expression of pro-inflammatory genes triggered by α-synuclein. In conclusion, we revealed novel roles for miR-335 in both microglia and neuronal cells that strongly halt the effects of classical inflammatory stimuli or LRRK2-Wt overexpression, thus attenuating chronic neuroinflammation.

## Introduction

Parkinson’s disease (PD) is the second most common neurodegenerative disorder worldwide, mainly instigated by dopaminergic neurodegeneration in the *substantia nigra pars compacta* (Poewe et al., 2017). The etiology of PD is complex and involves chronic neuroinflammation, mitochondrial dysfunction and oxidative stress (Poewe et al., 2017). Even though mostly sporadic, about 10% of all cases are currently estimated to be related to monogenic forms of PD (Henn et al., 2005; Poewe et al., 2017). Pathogenic mutations in the leucine-rich repeat kinase 2 (*LRRK2*) gene are the most frequent known cause of monogenic PD and are usually associated with a toxic gain-of-function of LRRK2 kinase activity (Zimprich et al., 2004; Healy et al., 2008). Importantly, the most frequent LRRK2 mutation, G2019S, can be relatively common depending on the ethnic group, with frequencies of 35.7% in sporadic and 42% in familial cases, in specific populations (Mata et al., 2006; Healy et al., 2008).

Although the role of LRRK2 is still not completely understood, LRRK2 pathogenic mutations are associated with dopaminergic neuronal cell death, inflammatory responses, and oxidative damage (Mata et al., 2006; Tsika and Moore, 2012). For instance, LRRK2 seems to be involved in the regulation of survival/inflammatory signaling pathways, such as mitogen-activated protein kinase (MAPK) pathways, whose activation may eventually lead to neuronal death (Chen et al., 2012). Interestingly, it has also been suggested that, in specific conditions, wild-type (wt) LRRK2 overexpression may protect SH-SY5Y cells from death, by selectively activating ERK1/2 signaling (Liou et al., 2008). Moreover, an exacerbation of LRRK2 levels in different immune cells, such as microglia or macrophages, has been reported in response to inflammatory stimuli, such as lipopolysaccharide (LPS) or interferon-γ (IFN-γ), thereby perpetuating inflammation (Gardet et al., 2010; Gillardon et al., 2012). The discoveries that both pharmacological and genetic inhibition of LRRK2 can be neuroprotective in preclinical models of PD (Chan and Tan, 2017; West, 2017; Zhao et al., 2017; Chen et al., 2018) have placed LRRK2 at the center of disease modifying PD strategies. In addition, recent findings also suggest that LRRK2 plays a role in the pathogenesis of PD, indicating that LRRK2-targeted therapies might, therefore, be beneficial in both subtypes of PD (Tolosa et al., 2020).

Throughout the years, several experimental models have been developed to mimic PD, including the systemic administration of animals with 6-hydroxydopamine (6-OHDA) and 1-methyl-1-4-phenyl-1,2,3,6-tetrahydripyridine hydrochloride (MPTP) (Dauer and Przedborski, 2003). However, the neurotoxin MPTP has been the most widely used to mimic PD-associated nigrostriatal degeneration, since it can be systemically administered and human exposure to MPTP induces severe parkinsonism (Meredith and Rademacher, 2011; Langston, 2017).

MicroRNA (miRNA or miR) dysregulation can also contribute to the development and progression of a wide variety of human diseases, including PD, where miRNAs have been associated with neuroinflammation (Martins et al., 2011; Miñones-Moyano et al., 2011; Patil et al., 2019). In this regard, miR-335 has recently been involved in PD. The results are somehow contradictory, with some authors suggesting that miR-335 is downregulated in peripheral blood mononuclear cells (PBMCs) and sera of PD patients, while others have found increased levels of miR-335 in PD serum samples (Yılmaz et al., 2016; Patil et al., 2019; Oliveira et al., 2020). Importantly, some authors also demonstrated that miR-335 upregulation reduces inflammation and reactive oxygen species (ROS) in a sepsis mouse model (Gao et al., 2018). In accordance, miR-335 downregulation appears to affect mitochondrial dynamics, autophagy and apoptosis in SH-SY5Y neuronal cells (De Luna et al., 2020). Interestingly, *in silico* and *in vitro* studies point LRRK2 mRNA as a target of this miRNA (Martins et al., 2011; Yılmaz et al., 2016; Patil et al., 2019; Oliveira et al., 2020).

Thus, our main hypothesis is that miR-335 regulates key inflammatory events by targeting LRRK2. In the present study, we demonstrated that miR-335 is reduced in experimental models of PD and in serum of idiopathic PD (iPD) and LRRK2-associated PD (LRRK2-PD) patients vs. healthy individuals, corroborating its clinical relevance during PD progression. In addition, miR-335 overexpression protected microglial cells from LPS-induced inflammation, by reducing RIP1 and RIP3 protein levels, proinflammatory cytokine expression and ERK1/2 activation. On a functional level, miR-335 directly targeted LRRK2 and reduced wild-type LRRK2-driven inflammation. The combination of novel miRNA strategies with LRRK2 inhibition may translate into promising and innovative therapeutic approaches to tackle PD.

## Materials and Methods

### Cell Culture and Reagents

The BV2 and N9 murine microglial cell lines, kindly provided by Elsa Rodrigues (University of Lisbon), were cultured in RPMI 1640 medium (GIBCO Life Technologies, Inc. Grand Island, United States), supplemented with 10% heat inactivated fetal bovine serum (FBS), 1% antibiotic/antimycotic solution and 1% GlutaMAX^TM^ (GIBCO). The SH-SY5Y human inducible WT α-synuclein (α-syn) cell line was cultured in RPMI 1640 medium, supplemented with 10% FBS, 1% penicillin (100 U/mL) (GIBCO), 100 mg/mL streptomycin (GIBCO), 250 μg/mL G418 (Thermo Fisher Scientific, Rockford, IL, United States) and 50 μg/mL hygromycin B (Thermo Fisher). α-synuclein expression was switched off by adding doxycycline (2 μg/mL) (Vekrellis et al., 2009). Cells were maintained at 37°C in a humidified atmosphere of 5% CO_2_. LPS was from *Escherichia coli* 055:B5 (#437625; Calbiochem, San Diego, CA, United States).

### MPTP Animal Model

Animal experiments were performed according to the animal welfare organ of the Faculty of Pharmacy, University of Lisbon, approved by the competent national authority *Direção-Geral de Alimentação e Veterinária* (DAGV) and in accordance with the EU Directive (2010/63/UE), Portuguese laws (DR 113/2013, 2880/2015, and 260/2016) and all relevant legislation. We performed a sub-acute MPTP mouse model in 13-week-old male C57BL/6N wild-type (Wt) obtained from the Charles River Laboratories (Wilmington, MA, United States). Mice were intraperitoneally (i.p.) injected with a single dose of MPTP-HCl (40 mg/kg; Sigma-Aldrich, St. Louis, MO, United States), dissolved in sterile 0.9% saline, or vehicle only (control group); seven animals per group were used (Saporito et al., 2000; Dionísio et al., 2019). After 30 days, mice were sacrificed in a CO_2_ chamber followed by transcardiac perfusion with ice-cold phosphate buffered saline (PBS). Serum was collected and stored at −80°C.

### miRNA Expression in Human Serum

We analyzed serum samples from 40 iPD, 41 LRRK2-PD patients and 40 control individuals with no known neurological disorder or family history of PD. Cases were selected from a randomized cohort of 867 iPD patients included at the Movement Disorders biobank (Instituto de Medicina Molecular, Lisbon, Portugal). Healthy controls were selected from a randomized cohort of 287 individuals of the same biobank. The LRRK2-PD group included 40 patients that carried the G2019S mutation and 5 patients that carried the R1441H mutation. All participants were recruited at the Movement Disorders outpatient clinic of the Hospital de Santa Maria (Lisbon, Portugal). Consent for inclusion in the study was obtained before participation and the study was performed in accordance with the Declaration of Helsinki and the protocol approved by the Ethics Committee of Hospital de Santa Maria. Serum isolation and miRNA extraction was performed as previously reported (Oliveira et al., 2020). miRNA expression was determined using TaqMan Universal Master Mix II no UNG (Thermo Fisher Scientific) and the 7500 Sequence Detection System (Applied Biosystems, Foster City, CA, United States), according to the manufacturer’s recommendations. Relative miR-335-3p expression levels of each subject were determined by the comparative ΔΔCt method using the spike-in cel-miR-39-3p (Thermo Fisher Scientific, Rockford, IL, United States) as the normalization control. miR-335 expression levels of each PD patient were normalized to the mean value of healthy controls.

### Cell Transfection

BV2, N9, and SH-SY5Y cells were transfected with 40 nM of a specific miR-335-3p precursor (pre-miR-335-3p; Ambion, Thermo Fisher Scientific, Inc.) or a pre-miR negative control (pre-miR-Control; Ambion, Thermo Fisher Scientific, Inc.) 24 h after plating. To evaluate the targeting of LRRK2 by miR-335-3p, BV2, and SH-SY5Y cells were co-transfected with 150 ng of a reporter plasmid driven by the SV40 basal promotor, harboring the LRRK2 3′ untranslated region (UTR) (HmiT002101-MT06, Tebu-bio, Lisbon, Portugal), or a negative control region (CmiT000001-MT06, Tebu-bio), upstream of the humanized firefly luciferase gene, in combination with the pre-miR-335-3p/pre-miR-Control or anti-miR-335-3p/anti-miR-Control (Ambion, Thermo Fisher Scientific, Inc.), for 24 h. For normalization, expression of the Renilla luciferase gene, contained in the reported plasmid, was used. Reporter assays were performed using Dual-Luciferase^®^ Reporter Assay (Promega Corp.), according to the manufacturer’s instructions. In LRRK2 overexpression experiments, BV2 or SH-SY5Y cells were transfected with 500 ng of pDEST53-LRRK2-WT DNA plasmid, gift from Mark Cookson (#25044, Addgene, Watertown, MA, EUA) (Greggio et al., 2006) or empty-vector for 24 h, before further treatments. Moreover, BV2 cells were transfected with 250 ng of a plasmid encoding a constitutively active form of mitogen-activated protein kinase (MEK1^∗^) (pCMB-deltaN3-MEK1), kindly provided by Dr. Roger J. Davis (Howard Hughes Medical Institute) or empty vector for 24 h before further treatments. All transfections were performed with Lipofectamine 3000^TM^ (Invitrogen, Thermo Fisher Scientific, Inc.), according to the manufacturer’s recommendations.

### Cell Viability/Death Assays

BV2 cells were plated in 96-well plates at 5 × 10^3^ cells/well and transfected the next day for 24 h before exposure to 100 ng/mL LPS for additional 24 h. SH-SY5Y cells, with or without overexpression of α-syn, were plated in 96-well plates at 4 × 10^4^ cells/well and transfected the next day for 24 h. Cellular metabolic activity was determined using CellTiter 96^®^ Aqueous Non-Radioactive Cell Proliferation (MTS) Assay (Promega, Madison, WI, United States). Alterations in absorbance were measured at 490 nm using GloMax^®^ Multi Detection System (Sunnyvale, CA, United States). Cell membrane integrity was determined using the lactate dehydrogenase (LDH) Cytotoxicity Kit^*PLUS*^ (Roche Diagnostics GmbH, Mannheim, Germany). Absorbance was measured at 490 nm, with 620 nm reference wavelengths, using a BioRad Model 680 microplate reader.

### Protein Extraction and Immunoblotting Analysis

BV2 and N9 cells were plated in 35-mm dishes at 1.1 × 10^5^ cells/dish and transfected the next day for 24 h before treatment with 100 ng/mL LPS for additional 24 h. SH-SY5Y cells, with or without overexpression of α-syn, were plated in 35-mm dishes at 12 × 10^5^ cells/dish and transfected the next day for 24 h. Cells were collected in nonyl phenoxypolyethoxylethanol (NP-40) lysis buffer [1% NP-40, 20 mM Tris–HCl pH 7.4, 150 mM NaCl, 5 mM EDTA, 10% glycerol, 1 mM dithiothreitol, and 1x Halt Protease and Phosphatase Inhibitor Cocktail EDTA-free (Pierce, Thermo Fisher Scientific, Rockford, IL, United States)], followed by sonication and centrifugation at 3,200 *g* for 10 min at 4°C. Total protein extracts were recovered and stored at −80°C. Protein concentration was calculated using the colorimetric Bradford method (Bio-Rad), according to the manufacturer’s recommendations. Equal amounts of protein (40 μg) were denatured and electrophoretically resolved on 6–8% SDS-polyacrylamide gels and transferred onto nitrocellulose membranes. Transient staining was performed with 0.2% Ponceau S (Merck, Darmstadt, Germany) to confirm protein loading and transfer. Membrane blocking was performed using 5% non-fat dried milk in Tris-buffered saline (TBS) for 1 h. Then, membranes were incubated overnight at 4°C with the following primary rabbit antibodies: RIP1 (#3493, Cell Signaling, MA, United States), RIP3 (#135170, Santa Cruz Biotechnology), p-MLKL (Ser358) (#196436, Abcam; Cambridge, Unite Kingdom), MLKL (#M6697, Sigma-Aldrich), IkB (#135170, Santa Cruz Biotechnologies), p-p38 (Thr180/Tyr182) (#9211, Cell Signaling), Erk1/2 (#4695, Cell Signaling), and with the following primary mouse monoclonal antibodies: JNK, p-JNK (Thr183/Tyr185), p38α/β, p-Erk1/2 (Tyr204) (#7345, #6254, #7972, #7383, Santa Cruz Biotechnologies) and p-IkB (Ser32/36) (#9246, Cell Signaling) and LRRK2 (#133474, Abcam) and finally with goat secondary antibodies conjugated with horseradish peroxidase anti-mouse or anti-rabbit (Bio-Rad Laboratories, Hercules, CA, United States) for 2 h at room temperature. Membranes were then processed for protein detection using Immobilon^TM^ Western (Merck Millipore, Burlington, MA, United States) or SuperSignal^TM^ West Femto Maximum Sensitivity Substrate (Pierce, Thermo Fisher Scientific). β-Actin (AC-15, Sigma Aldrich) was used as endogenous control. Densitometric analysis was performed with the Image Lab Software version 5.1 Beta (Bio-Rad).

### Quantitative Real Time-PCR (qRT-PCR)

BV2 and N9 cells were plated in 12-well plates at 4 × 10^4^ cells/well and transfected the next day for 24 h before treatment with 100 ng/mL LPS for additional 24 h. SH-SY5Y cells, with or without overexpression of α-syn, were plated in 12-well plates at 5 × 10^5^ cells/well and transfected in the following day for 24 h. Total RNA was extracted using TRIzol^TM^ reagent (Invitrogen, Grand Island, United States) and quantified using a Qubit^TM^ 2.0 fluorometer (Invitrogen). RNA was then converted into cDNA using NZY Reverse Transcriptase (NZYTech, Lisbon, Portugal). qRT-PCR was performed in the QuantStudio^TM^ 7 Flex Real-Time PCR System (Thermo Fisher Scientific Inc.). The following primer sequences were used: *COX2* gene, 5′-CAGCCAGGCAGCAAATCCTT (forward) and 5′-AGTCCGGGTACAGTCACACT (reverse); *HPRT* gene, 5′-GGTGAAAAGGACCTCTCGAAGTG (forward) and 5′-TA GTCAAGGGCATATCCAACAACA (reverse); *IL-1β* gene, 5′-TG CCACCTTTTGACAGTGATG (forward) and 5′-TGATGTGC TGCTGCGAGATT (reverse); *IL-6* gene, 5′-ATGAACTCCTTC TCCACAAGC (forward) and 5′-GTTTTCTGCCAGTGCCTGT TTG (reverse); *NLRP3* gene, 5′-GAGCCTACAGTTG GGTGAAATG (forward) and 5′-CCACGCCTACCAGGAAA TCTC (reverse); and *TNF-α* gene, 5′-AGGCACTCCCC CAAAAGATG (forward) and 5′-TGAGGGTCTGGGCCATA GAA (reverse). Two independent reactions for each primer set were performed in a final volume of 12.5 μL comprising 2x Power SYBR green PCR master mix (Thermo Fisher Scientific, Inc.) and 360 nM of each primer. The relative expression levels of each gene of interest were determined based on the standard curve normalized to the level of the housekeeping gene hypoxanthine-guanine phosphoribosyltransferase (*HPRT*). For miR-335-3p, TaqMan^®^ Gene Expression Assay (Thermo Fisher Scientific, Inc.) was used. U6 or cel-miR-39-3p were used as normalization control for cell extracts or serum samples, respectively. Relative amount of miR-335-3p was calculated by the threshold cycle (2^–ΔΔ*Ct*^) method.

### Statistical Analysis

Data analysis were performed with *t-*test and one-way analysis of variance (ANOVA) followed by *post hoc* Bonferroni’s test. Statistically significance was achieved when values of *p* < 0.05. Analysis and graphical presentation were presented with the GraphPad Prism software Version 8 (GraphPad Software Inc., San Diego, CA, United States). Results are showed as mean ± standard error of the mean (SEM).

## Results

### Patient Characterization

In this study, we included 40 iPD patients, 45 LRRK2-PD patients and 40 age- and gender-matched healthy controls. The major demographic and clinical features of patients and controls are presented in Table 1. Of note, patients covering the full spectrum of early to advanced PD, characterized by Hoehn and Yahr stage (1–5) were included. Further, at the time of sample collection, all patients were under treatment with antiparkinsonic medication. Age and gender equilibrium were assured between the three groups.

**TABLE 1:** Clinical features of patients and controls.

Patients characteristics	Controls (*n* = 40)	iPD (*n* = 40)	LRRK2-PD (*n* = 45)
Age (years)	67.4 ± 8.19	70.4 ± 10.2	70.0 ± 9.0
Gender (F/M)	20/20	20/20	31/14
Age at symptom onset (years)	–	58.2 ± 12.7	56.4 ± 11.9
Disease duration (years)	–	12.3 ± 9.1	13.6 ± 7.8
Hoehn and Yahr	–	2.5 ± 0.9	2.7 ± 1.0
Family history of PD (%)	–	35.0	63.4

*Data are presented as mean ± standard deviation. iPD, idiopathic Parkinson’s disease; LRRK2-PD, LRRK2 mutation Parkinson’s disease.*

### miR-335 Is Reduced in Experimental Models of PD and in the Sera of PD Patients

Recent studies have shown that the expression of miR-335 is altered in PD (Martins et al., 2011; Patil et al., 2019; Oliveira et al., 2020). Moreover, LRRK2 was pointed as a potential target of miR-335 (Martins et al., 2011). Here, we decided to further dissect the role of miR-335 in PD pathogenesis. We started by analyzing the expression pattern of miR-335 in several experimental models of PD. As an *in vitro* model of PD, we used the BV2 murine microglia cell line transiently transfected with a plasmid encoding wild-type LRRK2 (LRRK2-Wt), or empty vector, followed by LPS stimulation. Our results showed that LRRK2-Wt overexpression and/or cell incubation with LPS for 24 h significantly reduced miR-335 expression levels (Figure 1A). *In vivo*, we used 13-week-old male, injected intraperitoneally with a single dose of MPTP, or vehicle, and euthanized 30 days later, as a more clinically relevant model. This PD mouse model displays stable nigrostriatal dopaminergic neurodegeneration at 30 days, which is in accordance with the notion that dopaminergic neurodegeneration in PD patients majorly precedes the development of motor symptoms (Saporito et al., 2000; Kordower et al., 2013; Dionísio et al., 2019). We observed that MPTP-injected mice presented a significant reduction of miR-335 in the serum, when compared to control mice (Figure 1B). Finally, we determined the expression levels of miR-335 in serum samples of 40 iPD patients, 41 LRRK2-PD patients and 40 healthy controls, and confirmed that miR-335 was significantly reduced in the sera of iPD and LRRK2-PD patients in comparison with control subjects (Figure 1C). Although miR-335 levels were not significantly reduced in iPD patients in comparison with LRRK2-PD patients, a slight tendency of miR-335 to be reduced in iPD patients was observed, which could suggest that the role of LRRK2 in reducing miR-335 levels contributes to PD pathology in combination with several other mechanisms. Overall, these results indicate that miR-335 is reduced both *in vitro* and *in vivo* experimental models of PD, and most importantly, in the sera of PD patients, which highlights the potential of modulating miR-335 to alleviate PD pathogenesis.

**FIGURE 1:** miR-335 is reduced in *in vitro* and *in vivo* experimental models of PD and in the sera PD patients. **(A)** qRT-PCR analysis of miR-335 in BV2 microglial cells transfected with LRRK2-Wt overexpression plasmid, or empty vector, for 24 h and then stimulated with 100 ng/mL LPS for additional 24 h. **(B)** qRT-PCR analysis of miR-335 in the sera of MPTP-injected mice or control mice, euthanized at 30 days after MPTP injection. Values were normalized to the mean of control mice. **(C)** qRT-PCR analysis of miR-335 in serum of iPD and LRRK2-PD patients and control individuals. Values were normalized to the mean of control healthy individuals. Results are expressed as mean ± SEM. ^∗^*p* < 0.05 vs. Control; ^§^*p* < 0.05 vs. control Empty vector.

### miR-335 Overexpression Reduces LPS-Mediated RIP1 and RIP3 Increased Levels

Emerging evidence suggest a role of miR-335 in regulating inflammation in different experimental models of disease. Moreover, several authors have proposed that key necroptosis mediators such as RIP1 and RIP3 are involved in inflammatory responses, especially in macrophages and microglia, without necroptosis commitment (Christofferson et al., 2012; Ito et al., 2016; Ofengeim et al., 2017; Degterev et al., 2019). Here, to determine the involvement of RIP1 and RIP3 in the inflammatory response, we used BV2 and N9 microglia cells transfected with pre-miR-335, or pre-negative control (NC), for 24 h, followed by stimulation with LPS for additional 24 h; and SH-SY5Y neuroblastoma cells, with or without α-syn overexpression, transfected with pre-miR-335 or NC for 24 h. In both microglia and neuroblastoma cells, transfection with pre-miR-335 significantly increased miR-335 expression levels, thus confirming miRNA transfection efficiency (Supplementary Figures 1A,B). In addition, as expected, stimulation of BV2 cells with LPS or α-syn overexpression in SH-SY5Y cells did not induce cell death in MTS and LDH release assays (Supplementary Figures 1C,D). Similarly, miR-335 overexpression did not affect cell viability in both cell lines (Supplementary Figures 1C,D). However, LPS stimulation in BV2 and N9 cells significantly increased RIP1 and RIP3 protein levels, thus indicating that LPS-induced protein expression of RIP1 and RIP3 may be related to inflammatory events (Figures 2A,B). Importantly, miR-335 overexpression *per se* did not influence RIP1 and RIP3 levels, while concomitant LPS stimulation and miR-335 overexpression significantly reduced LPS-induced RIP1 and RIP3 protein expression, further suggesting a role for this miRNA in decreasing inflammation (Figures 2A,B). In agreement, a marker of necroptosis commitment such as the p-MLKL/MLKL ratio showed no significant differences (Figures 2A,B). Moreover, no differences were observed in RIP1 and RIP3 protein levels in BV2 cells overexpressing LRRK2-Wt (Supplementary Figure 2A). In SH-SY5Y cells with or without α-syn overexpression and/or miR-335 overexpression, no differences were observed in RIP1, RIP3, and MLKL protein levels (Supplementary Figure 2B).

**FIGURE 2:** Modulation of LPS-induced protein expression of RIP1 and RIP3 by miR-335. BV2 microglial cells **(A)** and N9 microglial cells **(B)** were transfected with pre-miR-335 or negative control (NC) for 24 h and then stimulated with LPS for additional 24 h. Total protein extracts were prepared for Western blot analysis of RIP1, RIP3, and p-MLKL/MLKL ratio. Representative immunoblots are presented. β-Actin was used as loading control. Values are expressed as mean ± SEM of three independent experiments. *p < 0.05 vs. NC; ^≠^*p* < 0.05 vs. NC exposed to LPS.

### miR-335 Overexpression Attenuates LPS- or α-Syn-Mediated Expression of Proinflammatory Mediators and LPS-Induced ERK1/2 Activation

Some authors have already proposed that miR-335 downregulation may have a deleterious effect by increasing the production of proinflammatory mediators in an inflammatory sepsis mouse model (Gao et al., 2018). To further determine the role of miR-335 in modulating inflammatory events, BV2 and N9 microglia cells were transfected with a pre-miR-335 or NC for 24 h, and further incubated with LPS for additional 24 h. Similarly, SH-SY5Y neuroblastoma cells with or without α-syn overexpression were transfected with a pre-miR-335 or NC for 24 h. Our results demonstrated that incubation of BV2 and N9 cells with LPS significantly increased TNF-α and IL-1β; or TNF-α, IL-1β, COX2, and NLRP3 mRNA levels, respectively (Figures 3A,B). No differences were observed in COX2 and NLRP3 mRNA levels in BV2 cells exposed to LPS (Figure 3A). As expected, miR-335 overexpression by itself did not influence mRNA levels of these cytokines. However, concomitant LPS incubation and miR-335 overexpression significantly decreased the mRNA levels of proinflammatory mediators (Figures 3A,B). In respect to neuronal cells, α-syn overexpression in SH-SY5Y cells significantly increased TNF-α and IL-6 mRNA levels, while no differences were observed in COX2, thereby indicating an α-syn-dependent inflammatory status in these cells (Figure 3C). Again, miR-335 overexpression alone did not influence the expression of these proinflammatory genes. However, when cells overexpress α-syn, miR-335 increased levels significantly attenuate α-syn-induced TNF-α and IL-6 (Figure 3C). These results confirm the potential of miR-335 in modulating inflammation in both neuronal and microglial cells.

**FIGURE 3:** Modulation of LPS or α-syn-mediated proinflammatory mRNA levels by miR-335. BV2 **(A)** and N9 **(B)** cells were transfected with a pre-miR-335 or pre-NC for 24 h, and then stimulated with LPS for additional 24 h. **(C)** SH-SY5Y cells with or without overexpression of α-syn were transfected with a pre-miR-335 or pre-NC for 24 h. mRNA levels were measured by qRT-PCR. Results are expressed as mean ± SEM from three independent experiments. ^≠^*p* < 0.01 vs. NC; *p < 0.05 vs. NC overexpressing α-syn or NC exposed to LPS.

Then, to further confirm mRNA proinflammatory gene expression and dissect inflammatory signaling pathways modulated by miR-335, we investigated the phosphorylation states of JNK (Thr183/Tyr185), p38 (Thr180/Tyr182), and ERK1/2 (Tyr204), three classic MAPK inflammatory signaling pathways, as well as NF-κB activation, which is a key mediator of inflammatory responses (Hashimoto et al., 2003; Tortarolo et al., 2003; Liu et al., 2017), in BV2 cells exposed to LPS from 30 min up to 24 h. As depicted in Figure 4, ERK1/2 pathway was activated at 4 and 6 h of LPS exposure (Figures 4A,B), but not at earlier or later time points (data not shown), as determined by the ratio between phosphorylated and total protein levels. Similarly, NF-κB was strongly activated at 4 and 6 h post LPS, as indirectly determined by the p-IκB/IκB ratio (Figures 4A,B). p38 and JNK pathways showed no alterations (Figure 4A). Importantly, transfection of cells with miR-335 alone did not activate these signaling pathways; however, miR-335 overexpression significantly reduced LPS-induced ERK1/2 and NF-κB activation (Figures 4A,B). To further confirm that the observed decrease in LPS-induced ERK1/2 levels is mediated by miR-335, we determined proinflammatory mRNA levels in BV2 cells after transfection with a plasmid encoding a constitutive active form of MEK1 (MEK1^∗^), which is the upstream kinase of ERK1/2. Our results showed that expression of MEK1^∗^ tended to abrogate miR-335 effect, as observed by an increase in TNF-α and IL-1β mRNA levels (Supplementary Figure 3).

**FIGURE 4:** Modulation of ERK1/2 and NF-κB activation by miR-335. BV2 cells were transfected with a pre-miR-335 or pre-NC for 24 h and then stimulated with LPS for 4 or 6 h. Representative immunoblots for p-ERK/ERK, p-JNK/JNK, p-p38/p38, and p-IκB/IκB ratios **(A)** and densitometric analysis of p-ERK/ERK and p-IκB/IκB ratios **(B)** are presented. Results are presented as mean ± SEM of three independent experiments. *p < 0.0.5 vs. C 0 h; ^≠^*p* < 0.05 vs. LPS 4 h; ¥*p* < 0.05 vs. LPS 6 h.

### miR-335 Directly Targets LRRK2 and Its Overexpression Attenuates LRRK2-Wt-Driven Inflammatory Events

Previous *in silico* studies have proposed LRRK2 as a putative target of miR-335, which was further confirmed *in vitro* (Yılmaz et al., 2016; Patil et al., 2019). Here, using dual-luciferase assay and western blot analysis, we also confirmed that miR-335 directly targets LRRK2 in both BV2 microglial and SH-SY5Y neuroblastoma cells (Figures 5A–D). In addition, using well-known *in silico* tools including TargetScan and PicTar databases, we found that α-syn 3′-UTR is also a putative target of miR-335 (Supplementary Figure 4). Although *LRRK2* pathogenic mutations are linked to dopaminergic cell death, there is also evidence suggesting that LRRK2-Wt overexpression upregulates α-syn levels, thereby influencing the pathological output of LRRK2-related PD (Lin et al., 2009; Carballo-Carbajal et al., 2010). Here, we used BV2 microglial cells co-transfected with LRRK2-Wt expression plasmid and pre-miR-335, and further incubated with LPS for additional 24 h; and SH-SY5Y neuroblastoma cells, with or without α-syn overexpression co-transfected with LRRK2-Wt and pre-miR-335. Transfection of BV2 cells with LRRK2-Wt plasmid resulted in a significant increase of LRRK2 protein, which in turn was attenuated by miR-335 overexpression (Figure 5D). Additionally, LRRK2-Wt overexpression, with or without concomitant LPS incubation, did not affect cell viability, as observed by MTS and LDH assays (Supplementary Figure 5A). Also, miR-335 overexpression did not induce any alteration in cell viability, in the presence or absence of LRRK2-Wt overexpression (Supplementary Figure 5A). Similar results were observed in SH-SY5Y cells with or without α-syn and concomitant overexpression of LRRK2-Wt (Supplementary Figure 5B).

**FIGURE 5:** MiR-335 directly targets LRRK2. **(A)** SH-SY5Y cells were co-transfected with a LRRK2 luciferase reporter vector, or negative control, and pre-miR-335/pre-NC; or anti-miR-335/anti-NC for 24 h. **(B)** BV2 cells were co-transfected with a LRRK2 luciferase reporter vector, or negative control, and pre-miR-335/pre-NC; or anti-miR-335/anti-NC for 24 h. Renilla luciferase signal was used as an internal standard control. Results are presented as mean ± SEM of three independent experiments. *p < 0.0.5 vs. pre-NC. **(C)** Representative immunoblots are presented for LRRK2 in SH-SY5Y cells. β-Actin was used as loading control. **(D)** BV2 cells were co-transfected with a LRRK2-Wt or empty vector plasmid and with a pre-miR-335 or pre-NC for 24 h, and then stimulated with LPS for additional 24 h. Representative immunoblots are presented for LRRK2. β-Actin was used as loading control. **(E)** Modulation of LRRK2-Wt-induced proinflammatory mRNA levels by miR-335. BV2 cells were co-transfected with a LRRK2-Wt or empty vector plasmid and with a pre-miR-335 or pre-NC for 24 h, and then stimulated with LPS for additional 24 h. TNF-α, IL-1β, COX2, and NLRP3 mRNA levels were measured by qRT-PCR. Results are expressed as mean ± SEM from three independent experiments. *p < 0.05 vs. empty vector; ^≠^*p* < 0.05 vs. empty vector transfected with pre-NC, ^¶^ *p* < 0.05 vs. LRRK2-Wt; ^§^ *p* < 0.05 vs. LRRK2-Wt exposed to LPS. **(F)** Modulation of LRRK2-Wt-induced proinflammatory mRNA levels by miR-335. SH-SY5Y cells with or without overexpression of α-syn were co-transfected with a LRRK2-Wt or empty vector plasmid and with a pre-miR-335 or pre-NC for 24 h. TNF-α, IL-1β, and COX2 mRNA levels were measured by qRT-PCR. Results are expressed as mean ± SEM from three independent experiments. *p < 0.05 vs. empty vector; *p* < 0.05 vs. empty vector transfected with pre-NC, **p < 0.05 vs. NC overexpressing α-syn; ^¶^ *p* < 0.05 vs. LRRK2-Wt without α-syn overexpression; ^§^ *p* < 0.05 vs. LRRK2-Wt with α-syn overexpression.

Finally, the role of LRRK2 in inflammation has been studied since the identification of *LRRK2* as one of the genes causing susceptibility for the development of inflammatory diseases. Moreover, recent evidence shows that LRRK2 is elevated in immune cells, including microglia, where it may promote inflammation (Gillardon et al., 2012; Moehle et al., 2012). Thus, we wanted to explore whether LRRK2-Wt overexpression could influence the expression of proinflammatory genes, which may in turn be modulated by miR-335. We used BV2 microglia cells co-transfected with LRRK2-Wt or empty vector plasmid and pre-miR-335 for 24 h, and further incubated with LPS for additional 24 h, or SH-SY5Y cells overexpressing α-syn co-transfected with LRRK2-Wt or empty vector plasmid and pre-miR-335 for 24 h. Here, LRRK2-Wt overexpression significantly increased TNF-α, IL-1β and NLRP3 but not COX2 mRNA levels. Concomitant treatment with LPS further increased the levels of these proinflammatory markers (Figure 5E). Importantly, miR-335 overexpression significantly reduced TNF-α and IL-1β mRNA levels in both LRRK2-Wt and LRRK2-Wt exposed to LPS conditions (Figure 5E). Similar results were observed in SH-SY5Y cells, where LRRK2-Wt overexpression significantly increased TNF-α, IL-1β and COX2 mRNA levels with or without α-syn overexpression (Figure 5F). More importantly, miR-335 overexpression also significantly decreased TNF-α and IL-1β mRNA levels (Figure 5F). These results confirm the role of miR-335 in protecting microglia and neuronal cells from an inflammatory phenotype.

## Discussion

In this study, we hypothesized that miR-335 plays important roles during inflammation by targeting LRRK2. We first determined the levels of miR-335 in different *in vitro* models and its circulating levels in *in vivo* PD-mimicking experimental models and in PD patients. Recent studies have shown that miR-335 may be linked to PD pathogenesis, since we and others have found reduced expression levels in whole blood, PBMCs and serum of PD patients compared with control subjects (Martins et al., 2011; Yılmaz et al., 2016; Oliveira et al., 2020). In accordance, here we observed that miR-335 is significantly reduced in the sera of both iPD and LRRK2-PD patients as compared with control subjects. Others have suggested that the role of miR-335 in PD pathogenesis is mediated by LRRK2 (Yılmaz et al., 2016; Patil et al., 2019). In this regard, we confirmed that miR-335 directly targets LRRK2 in BV2 and SH-SY5Y cells. Moreover, it has been demonstrated that LRRK2 expression is induced by inflammatory stimuli, such as LPS or IFN-γ in activated microglia, PBMCs and cultured bone marrow-derived macrophages (Gardet et al., 2010; Hakimi et al., 2011; Moehle et al., 2012). LRRK2 protein activation is linked to inflammatory signaling, while no significant differences occur in LRRK2 mRNA levels, which could suggest a post-transcriptional regulation, for instance by miRNAs (Moehle et al., 2012). Here, we showed that BV2 microglial cells stimulated with LPS presented a significant reduction in miR-335 expression levels. Moreover, concomitant overexpression of LRRK2-Wt also contributed to a reduction in the levels of this miRNA, which could indicate a feedback loop where an inflammatory stimulus reduces miR-335 expression, which may in turn promote an increase in LRRK2 protein levels, therefore exacerbating inflammation. In fact, others have shown that in response to TLR4 activation, LRRK2 inhibition, either by small-molecule kinase inhibitors or LRRK2 knockdown, reduces proinflammatory signaling pathways (Moehle et al., 2012). Furthermore, we determined miR-335 expression levels in the sera of mice subjected to a single injection of the MPTP neurotoxin, a well-known trigger of PD-related pathology, and observed that miR-335 was significantly reduced in these mice in comparison with control mice, which may suggest an overall reduction in miR-335 levels in the presence of an inflammatory environment. Indeed, others have demonstrated that MPTP-treated mice present increased expression of TLR4, which is involved in the release of proinflammatory molecules from microglia (Lofrumento et al., 2011; Shao et al., 2019). Overall, these results suggest that the levels of miR-335 decrease in response to inflammatory environments. Thus, it is possible to speculate about the potential role of this miRNA in contributing to an overall reduction of inflammation in animal models of PD-related pathologies.

Considering that miR-335 is reduced in different inflammatory PD models, we tested if elevating the levels of miR-335 could impact on inflammation. Notably, we observed that miR-335 overexpression significantly reduced RIP1 and RIP3 protein levels induced by LPS stimulation in BV2 and N9 microglial cells, while no differences were observed in p-MLKL/MLKL ratio nor in cell viability, indicating that modulation of RIP1/3 by miR-335 did not influence cell death by necroptosis in these models. In fact, some studies have demonstrated that proinflammatory stimulation of macrophages and microglia and consequent RIP1 activation, with or without RIP3 recruitment, could induce the expression of proinflammatory genes, with no MLKL involvement or cell death associated (Christofferson et al., 2012; Ito et al., 2016; Ofengeim et al., 2017; Degterev et al., 2019). Interestingly, no differences in RIP1 and RIP3 were observed in SH-SY5Y cells overexpressing α-syn, thus suggesting that, at least in our conditions, α-syn overexpression is not sufficient for inducing inflammatory-dependent activation of RIP1 and RIP3, or that the cells themselves may not rely as strongly on RIP1/3 signaling as microglial cells. Importantly, LPS stimulation of BV2 and N9 microglial cells as well as α-syn overexpression in SH-SY5Y cells strongly induced the expression of several proinflammatory genes, including TNF-α, IL-1β, IL-6, COX2, and NLRP3, which was counteracted by miR-335 overexpression, thus highlighting the role of miR-335 as an anti-inflammatory miRNA. These results are in accordance with other studies where miR-335 upregulation was associated with decreased inflammation through the reduction of proinflammatory gene expression, ROS levels and inflammasome activation in a sepsis mice model (Gao et al., 2018). In SH-SY5Y cells, others also demonstrated that miR-335 inhibition results in increased ROS production (De Luna et al., 2020).

Throughout the years, several lines of evidence have proposed that increased proinflammatory gene expression depends on the activation of multiple MAPKs, specially p38, ERK1/2 and JNK, and downstream activation of transcription factors, such as NF-κB. However, the precise mechanisms connecting these events to RIP1 and/or RIP3 activation are still poorly understood (Christofferson et al., 2012; Ito et al., 2016; Zhu et al., 2018). Interestingly, some studies demonstrated that increased LRRK2 protein levels promote ERK1/2 activation, without affecting p38 or JNK signaling pathways (Carballo-Carbajal et al., 2010). Our results are in accordance with these studies since miR-335 overexpression reduced LPS-induced ERK1/2 activation, thereby confirming its role in reducing inflammation which is probably mediated by LRRK2 inhibition. Overall, we observed that stimulation of cells with a proinflammatory stimulus, such as LPS, strongly increases RIP1 and RIP3 protein levels, which may consequently contribute to the activation of ERK1/2 pathway, thus leading to the downstream activation of NF-κB transcription factor, which may contribute to the induction of proinflammatory gene expression (Festjens et al., 2007; Humphries et al., 2015). Importantly, miR-335 demonstrated high anti-inflammatory potential by reducing these inflammatory mechanisms.

After determining the role of miR-335 overexpression in diminishing inflammation mediated by a classical inflammatory stimulus, we hypothesized that miR-335 could also reduce LRRK2-Wt-driven inflammation and/or cell death. LRRK2 has been widely described in the regulation of several inflammatory pathways and its activation associated with neuronal death (Chen et al., 2012). Interestingly, although LRRK2 mutations are commonly linked to neuronal death exacerbation, the role of LRRK2-Wt overexpression is not completely understood, with some studies showing a role in protecting SH-SY5Y cells from death (Liou et al., 2008), and others indicating a deleterious effect by increasing α-syn levels in HEK293 cells (Carballo-Carbajal et al., 2010). Moreover, in both SH-SY5Y and immune cells, LRRK2-Wt overexpression seems to have other detrimental effects, including mitochondrial fragmentation and inflammation (Marker et al., 2012; Moehle et al., 2012; Wang et al., 2012; Berwick et al., 2019). Our results showed that LRRK2-Wt overexpression did not induce cell death in BV2 nor SH-SY5Y cells. However, LRRK2-Wt overexpression strongly induced proinflammatory gene expression in BV2 microglia and SH-SY5Y neuroblastoma cells, while miR-335 overexpression attenuated this effect.

In conclusion, we have unraveled a novel role for miR-335 during inflammation in PD-like conditions in both microglial and neuronal cells, which are probably but not exclusively dependent on LRRK2 targeting. Here, miR-335 showed to be reduced in different *in vitro* and *in vivo* PD-mimicking models and in PD patients, while its overexpression strongly reduced inflammation induced by either LPS stimulation or LRRK2-Wt overexpression. These observations suggest that miR-335 overexpression may contribute to a less pro-inflammatory activation in PD, thereby contributing to attenuate chronic neuroinflammation and PD progression.

## Data Availability Statement

The raw data supporting the conclusions of this article will be made available by the authors, without undue reservation.

## Ethics Statement

The studies involving human participants were reviewed and approved by Ethics Committee of Hospital de Santa Maria, Lisbon, Portugal. The patients/participants provided their written informed consent to participate in this study. The animal study was reviewed and approved by Animal welfare, Faculty of Pharmacy, University of Lisbon, and approved by the competent national authority Direção-Geral de Alimentação e Veterinária (DAGV).

## Author Contributions

PD, JA, and CR: conceptualization. SO and LC: data curation. SO and PD: formal analysis. CR: funding acquisition. SO, PD, LC, MG, MC, MR, and JF: investigation. SO, PD, and MG: methodology. JA and CR: project administration. JA, JF, and CR: supervision. SO: writing—original draft. SO, PD, MG, LC, MC, MR, JA, JF, and CR: writing—review and editing. All authors have read and agreed to the published version of the manuscript.

## Conflict of Interest

The authors declare that the research was conducted in the absence of any commercial or financial relationships that could be construed as a potential conflict of interest.
